The article "Resveratrol Improves Mitochondrial Biogenesis Function and Activates PGC-1α Pathway in a Preclinical Model of Early Brain Injury Following Subarachnoid Hemorrhage" was retracted in 2025. Reason: concerns about the images.

# Resveratrol Improves Mitochondrial Biogenesis Function and Activates PGC-1α Pathway in a Preclinical Model of Early Brain Injury Following Subarachnoid Hemorrhage

**DOI:** 10.3389/fmolb.2021.620683

**Published:** 2021-04-22

**Authors:** Jian Zhou, Zaijia Yang, Ruiming Shen, Wangwang Zhong, Huiduan Zheng, Zhenggang Chen, Jianjian Tang, Juan Zhu

**Affiliations:** ^1^Department of Neurosurgery, The First Affiliated Hospital of Hainan Medical University, Haikou, China; ^2^School of Medical Management, Hainan Medical University, Haikou, China; ^3^Department of Rheumatology, The First Affiliated Hospital of Hainan Medical University, Haikou, China; ^4^Department of Neurology, Hainan Provincial People’s Hospital, Haikou, China; ^5^Hainan Provincial Key Laboratory for Human Reproductive Medicine and Genetic Research, Department of Reproductive Medicine, The First Affiliated Hospital of Hainan Medical University, Haikou, China

**Keywords:** subarachnoid hemorrhage, early brain injury, resveratrol, PGC-1α, mitochondrial biogenesis-function

## Abstract

Peroxisome proliferator-activated receptor gamma coactivator 1-alpha (PGC-1α) has been shown to play a pivotal role in the regulation of mitochondrial biogenesis in diseases. Resveratrol (RSV), a natural polyphenolic reagent, has powerful antioxidant properties and the ability to scavenge mitochondrial reactive oxygen species (ROS) in a variety of central nervous system diseases. However, the underlying molecular mechanisms of RSV on mitochondrial biogenesis in early brain injury (EBI) following subarachnoid hemorrhage (SAH) remain poorly understood. This study aimed to explore the potential neuroprotective effects of RSV on mitochondrial biogenesis and function by activation of the PGC-1α signaling pathway in a prechiasmatic cistern SAH model. PGC-1α expression and related mitochondrial biogenesis were detected. Amounts of nuclear respiratory factor 1 (NRF1) and mitochondrial transcription factor A (TFAM) were determined to evaluate the extent of mitochondrial biogenesis. Increased PGC-1α and mitochondrial biogenesis after SAH were observed in the temporal cortex. Resveratrol increased the expression of PGC-1α, NRF1, and TFAM, and promoted PGC-1α nuclear translocation. Moreover, RSV could scavenge excess ROS, increase the activity of superoxide dismutase (SOD), enhance the potential of mitochondrial membrane and ATP levels, reduce the number of mitochondrial DNA copy, and decrease the level of malondialdehyde (MDA). RSV significantly ameliorated the release of apoptosis-related cytokines, namely P53, cleaved caspase-3, cytochrome c, and BAX, leading to the amelioration of neuronal apoptosis, brain edema, and neurological impairment 24 h after SAH. These results indicate that resveratrol promotes mitochondrial biogenesis and function by activation of the PGC-1α signaling pathway in EBI following SAH.

The article "Resveratrol Improves Mitochondrial Biogenesis Function and Activates PGC-1α Pathway in a Preclinical Model of Early Brain Injury Following Subarachnoid Hemorrhage" was retracted in 2025. Reason: concerns about the images.

## Highlights

- RSV attenuated the mitochondria-dependent apoptosis following SAH.
- RSV reduced redundant ROS production induced by SAH.
- RSV activated the PGC-1α signaling pathway and promoted the modulation of PGC-1α nuclear shuttling following SAH.
- RSV ameliorated SAH-induced oxidative damage, brain edema, and neurological impairment.
- RSV could promote mitochondrial biogenesis-function against SAH-induced oxidative stress and apoptosis.

## Introduction

Subarachnoid hemorrhage (SAH) is a fatal cerebrovascular disease with high rates of morbidity and mortality. Accumulating evidence indicates that early brain injury (EBI) is the major cause of deterioration in patients with SAH. Therefore, treatment of EBI has been believed to be the principal target for patients with the disease. Studies have indicated that numerous pathophysiological processes are involved in the pathogenesis of EBI, such as mitochondrial dysfunction, oxidative stress, apoptosis, inflammation, autophagy, and brain edema (Fujii et al., 2013). Among them, mitochondrial dysfunction plays a pivotal role in EBI. Hence, improvement of mitochondrial dysfunction may be a promising therapeutic strategy for the treatment of EBI following SAH.

Mitochondria play a fundamental role in cellular homeostasis. A recent analysis indicated that mitochondrial dysfunction increases oxidative stress. Excessive reactive oxygen species (ROS) production contributes to oxidative damage, causing persistent injury to brain tissues after SAH. However, superfluous generation of ROS induced by SAH can lead to exhaustion of innate antioxidation and disturbance of the redox system, resulting in severe complications. Brain tissue is more susceptible to free radical attacks, leading to mitochondrial dysfunction, ultimately triggering the cascade of cell apoptosis involving P53, the Bcl-2 family, cytochrome c, and caspase-3, which induces lipid peroxidation, nucleic acid oxidation, and DNA breakdown (Shen et al., 2019). Therefore, reversal of mitochondrial dysfunction and promotion of mitochondrial biogenesis after SAH can improve mitochondrial function and maintain cell homeostasis. However, the exact underlying mechanisms of these processes have not yet been investigated in SAH. Mitochondria, especially mitochondrial DNA (mtDNA), are affected by ROS, and this may be modulated by the peroxisome proliferator-activated receptor (PPAR) γ coactivator-1 (PGC-1) family of transcriptional coactivators; also, they are susceptible to oxidative impairment. PGC-1α, a transcriptional coactivator of mitochondrial biogenesis that directly links external physiological stress to the regulation of mitochondrial biogenesis and function, is involved in energy homeostasis and metabolism.

The article "Resveratrol Improves Mitochondrial Biogenesis Function and Activates PGC-1α Pathway in a Preclinical Model of Early Brain Injury Following Subarachnoid Hemorrhage" was retracted in 2025. Reason: concerns about the images.

Resveratrol (RSV) is a polyphenolic compound with pleiotropic properties produced in a variety of plant species, such as red grapes, mulberries, peanuts, and wines. RSV eliminates excessive ROS when cellular homeostasis is disturbed. Recent studies have indicated beneficial effects of RSV, namely, anti-apoptotic, anti-inflammatory, and antioxidant activities (Zhou X. M. et al., 2014; Narayanan et al., 2015; Tellone et al., 2015; Hoda et al., 2017; Gomes et al., 2018). It has been shown that RSV can cross the blood–brain barrier (BBB) and be used to treat neuroinflammatory and neurodegenerative diseases (Li et al., 2014; Shao et al., 2014; Lopez et al., 2015). Several studies have indicated that RSV could regulate mitochondrial ROS homeostasis and enhance PGC-1α expression (Zhou X. et al., 2014). RSV can abrogate cardiac oxidative stress and mitochondrial dysfunction in diabetes (Mohammadshahi et al., 2014; Bagul et al., 2015; Wu et al., 2016). Various studies demonstrate that RSV can improve the activation of PGC-1α and its downstream signaling pathways (de Oliveira et al., 2016). However, the exact mechanisms by which RSV regulates mitochondrial biogenesis and function in SAH have not been fully elucidated. Thus, we conducted this study to confirm the hypothesis that RSV could exert a neuroprotective effect by improving mitochondrial biogenesis and function, *via* activation of the PGC-1α signaling pathway.

## Materials and Methods

### Animal Ethical Approval

Adult male Sprague–Dawley rats weighing 270 to 320 g were used in the study. The rats were maintained under standard conditions of temperature (22 ± 1°C), relative humidity (30%), and lighting (a 12/12-h light/dark cycle). Drinking water and food were given *ad libitum*. All experimental procedures and protocols were conducted by the Animal Care and Use Committee of Hainan Medical University (Haikou, China) and conformed to the Guide for the Care and Use of Laboratory Animals set by the National Institutes of Health (NIH).

### Subarachnoid Hemorrhage Model

The experimental SAH model in this study was produced as previously described (Wang et al., 2012). Briefly, rats were anesthetized using inhalation anesthesia with isoflurane (2% in oxygen gas, 300 ml/min) and subsequently placed in a stereotactic frame. Under stereotactic guidance, fresh autologous non-heparinized arterial blood (0.3 ml) from the femoral artery was injected aseptically into the prechiasmatic cistern of rats in 20 s with a syringe pump. The wound was then sutured. The sham group was injected with 0.3 ml artificial cerebrospinal fluid. The animals were allowed to recover in a head-down prone position for 45 min post SAH. After surgery, all the animals were returned to their cages, and food and water were supplied freely.

The article "Resveratrol Improves Mitochondrial Biogenesis Function and Activates PGC-1α Pathway in a Preclinical Model of Early Brain Injury Following Subarachnoid Hemorrhage" was retracted in 2025. Reason: concerns about the images.

The grade of SAH was blindly assessed with a grading system before euthanasia, as previously described (Sugawara et al., 2008). Rats with a grade of less than eight were excluded for having no obvious brain damage.

### Experimental Design

Rats were randomly assigned to one of the following groups: Sham, SAH, SAH + vehicle (SAH + V), and SAH + resveratrol (SAH + RSV). Resveratrol (Sigma-Aldrich, St. Louis, United States) was dissolved in an equal amount of DMSO solution (1% dimethyl sulfoxide in 0.9% saline) just before injection. Rats in the SAH + RSV group were treated with an intraperitoneal injection of 60 mg/kg resveratrol 2 and 12 h post SAH (Zhang et al., 2016a). Rats in the SAH vehicle-treated group were injected equal volumes of the vehicle at the corresponding time point. All the animals were euthanized 24 h post SAH (Zhou X. M. et al., 2014; Zhang et al., 2016b).

### Neurobehavioral Evaluation and Brain Water Content

The neurological scores was performed 24 and 72 h after SAH using a scoring methodology for appetite, activity, and neurologic deficits (Wang et al., 2012). All neurobehavioral evaluations were conducted by two veterinarians who were blind to the grouping.

Brain water content was measured by a wet/dry ration method (Xu et al., 2013). In brief, the brain of a rat was quickly obtained 24 h after SAH, and temporal cortical tissues were weighed immediately to acquire wet weight (WW). Brain samples were dried for 72 h at 80°C and weighed to obtain dry weight (DW). Brain water content was calculated as [(WW–DW)/WW] × 100%.

### Tissue Processing

The rats were sacrificed 24 h after SAH and perfused transcardially with phosphate-buffered saline (PBS). The same part of the inferior basal temporal lobe was harvested (Figure 1A). Then, the brain samples were analyzed for water content, Western blot, and biochemistry indexes. For immunofluorescence analysis and terminal deoxynucleotidyl transferase dUTP nick end labeling (TUNEL) staining, whole brain tissues were harvested then immersed in 4% buffered paraformaldehyde overnight.

**FIGURE 1:** Effects of RSV on subarachnoid hemorrhage (SAH) in rats. **(A)** Schematic representation of the inferior temporal cortex area sampled for analysis. **(B)** SAH grades. **(C)** Neurological function was assessed by neurological scores 24 and 72 h after SAH. **(D)** Brain water content in the RSV-treated group was obviously lower than that in the vehicle-treated group following SAH. Data were represented as mean ± SEM (*n* = 6). *p < 0.05, **p < 0.01, and ***p < 0.001 vs. sham group; ^ns^*p* > 0.05 vs. group with SAH, ^@^*p* > 0.05, ^#^*p* < 0.05, and ^##^*p* < 0.01 vs. vehicle-treated group.

The article "Resveratrol Improves Mitochondrial Biogenesis Function and Activates PGC-1α Pathway in a Preclinical Model of Early Brain Injury Following Subarachnoid Hemorrhage" was retracted in 2025. Reason: concerns about the images.

### Isolation of Mitochondria

Mitochondria from the inferior basal temporal lobe were extracted following the instructions of the manufacturer with the use of the Mitochondrial Isolation Kit for Tissue (Beyotime Institute of Biotechnology, Nantong, China). In brief, the temporal lobe was grounded in an ice-cold isolation buffer and then centrifuged at 1,200 × *g* for 3 min. The supernatants were collected and centrifuged at 14,000 × *g* for 14 min at 4°C to precipitate the mitochondria.

### Terminal Deoxynucleotidyl Transferase-Mediated dUTP Nick End Labeling Staining

Terminal deoxynucleotidyl transferase dUTP nick end labeling staining was determined using a TUNEL detection kit (ISCDD, Boehringer Mannheim, Germany) according to the instructions of the manufacturer. Quantitative analysis of TUNEL-positive cells in the temporal cortex was performed in six random non-overlapping fields (400×) under epifluorescence microscopy. The extent of brain injury was assessed using the apoptotic index, which is defined as the average number of TUNEL-positive neurons in each section. The positive cells were analyzed by two investigators who were blind to the grouping.

### Western Blot Analysis

Protein extraction was performed using the Total Protein Extraction Kit, Nuclear/Cytosol Extraction Kit, and Tissue Mitochondria Isolation Kit (Beyotime Biotech, Nantong, China) in accordance with the protocol provided by the manufacturer. Protein concentration was determined using the Bradford method. Protein samples (50 μg/lane) were separated on a 12% sodium dodecyl sulfate–polyacrylamide gel and electrophoretically transferred to polyvinylidene difluoride (PVDF) membranes. The membranes were blocked with 5% skim milk for 2 h at room temperature and then incubated overnight at 4°C with appropriate primary antibody using the following dilution ratio: P53 (1:400, Cell Signaling Technology (CST), Danvers, MA, United States), PGC-1α (1:1,000, CST, Danvers, MA, United States), NRF1 (1:1,000, CST, Danvers, MA, United States), TFAM (1:1,000, CST, Danvers, MA, United States), cytochrome c (1:1,000, Abcam, Cambridge, United Kingdom), Bax (1:200, Santa Cruz Biotechnology, Dallas, TX, United States), Bcl2 (1:200, Santa Cruz Biotechnology, Dallas, TX, United States), COX IV (1:1,000, CST, Danvers, MA, United States), H3 (1:1,000, CST, Danvers, MA, United States), β-actin (1:5,000, Bioworld Technology, Inc., Bloomington, MN, United States), and cleaved caspase-3 (1:1,000, CST, Danvers, MA, United States). Subsequently, the membranes were incubated with horseradish peroxidase-linked IgG for 2 h. Protein bands were visualized by enhanced chemiluminescence (ECL) Western blot detection reagents (Millipore, Billerica, MA, United States). Band relative density was evaluated using the ImageJ software.

The article "Resveratrol Improves Mitochondrial Biogenesis Function and Activates PGC-1α Pathway in a Preclinical Model of Early Brain Injury Following Subarachnoid Hemorrhage" was retracted in 2025. Reason: concerns about the images.

### Immunofluorescence Staining

Immunofluorescence staining was conducted according to the procedures of a previous immunostaining protocol as follows: briefly, sections (6 μm) were incubated in blocking buffer (5% normal fetal bovine serum in PBS containing 0.1% Triton X-100) for 2 h followed by overnight incubation with primary antibody at 4°C. Then, the sections were washed three times for 10-min with PBS and incubated with proper secondary antibodies for 1 h at room temperature. After the sections were again washed with PBS n, they were counterstained with DAPI, 4′,6-diamidino-2-phenylindole (1:1,000, Sigma-Aldrich, St. Louis, United States) for 2 min. After the sections were washed with PBS, they were cover slipped with an anti-fade mounting medium. Fluorescence microscopy imaging was conducted using a ZEISS HB050 inverted microscope system and analyzed using the Image-Pro Plus 6.0 software (Media Cybernetics, Rockville, MD, United States). All the brain sections were evaluated in six temporal cortical microscopic fields (400×) by two investigators who were blind to the experiment.

### Reactive Oxygen Species Content

Intracellular ROS contents were determined using the fluorescence probe dihydroethidium (DHE) according to the instructions of the manufacturer (Sigma-Aldrich, St. Louis, MO, United States). Briefly, the frozen sections were incubated in DHE and then treated with PBS for 30 min at 37°C in the dark. The sections were washed three times for 5 min in PBS (pH 7.4). Immunofluorescence imaging was performed using a ZEISS HB050 inverted microscope system. DHE-fluorescence intensity (representing the intracellular ROS levels) was measured using the Image-Pro Plus 6.0 software.

Production of mitochondrial ROS was detected using a MitoSOX^TM^ Red mitochondrial superoxide indicator (Thermo Fisher Scientific, Waltham, MA, United States). Fresh temporal cortex tissues weighing 10 mg were dispersed to single-cell suspension using a pipettor. The cells were washed twice with PBS and diluted in 5 mM MitoSOX^TM^ reagent stock solution in HBSS/Ca/Mg buffer to make a 5 μm MitoSOX reagent working solution. A working solution of 1.0 ml 5 μm MitoSOX reagent was applied to incubate the cells for 10 min at 37°C in the dark. Fluorescence was detected using a microplate reader at an emission wavelength of 510 nm and an excitation wavelength of 580 nm.

The article "Resveratrol Improves Mitochondrial Biogenesis Function and Activates PGC-1α Pathway in a Preclinical Model of Early Brain Injury Following Subarachnoid Hemorrhage" was retracted in 2025. Reason: concerns about the images.

### Nissl Staining

Nissl staining of the sections of paraffin-embedded brain tissues (5-μm thick) were conducted using cresyl violet and according to a previous study (Zhuang et al., 2012). Normal neurons have a relatively big cell body, rich incytoplasm, with one or two big round nuclei. On the contrary, positive cells had irregular neuronal cell bodies, shrunken and hyperchromatic nuclei, and dried-up cytoplasm with vacuoles. Then, histological examination was performed by two investigators who were blind to the experiment to evaluate the ratio of positive cells.

### Mitochondrial MDA and SOD Content

Brain tissues were homogenized in 2 ml 10 mM PBS (pH 7.4). Following centrifugation at 12,000 × *g* for 20 min, the contents of mitochondrial MDA and SOD in the supernatant were quantitated spectrophotometrically according to the instructions of the manufacturer. Protein concentrations were determined using the Bradford method.

### Quantification of mtDNA

Total mtDNA was extracted from the inferior basal temporal lobe using a rapid animal genomic DNA isolation kit according to the instructions of the manufacturer. The mtDNA copy number was determined by the SYBR Green Quantitative RT-PCR kit (Sigma–Aldrich, St. Louis, United States) using specific primers for the mtDNA-coded NADH-dehydrogenase subunit 1 (ND1) gene and the nuclear DNA coded β-globin gene. The primer sequences are as follows:

ND1: forward: 5′–TCGACGTTAAAGCCTGAGACT–3′,
Reverse: 5′–TTAATCCCCGCCTGACCAATA–3′.
β-globin: forward 5′–GTCTACCCTTGGACCCAGAG–3′,
Reverse 5′–CCAAGTGTTTCAGGCCATCA–3′.
Relative transcript abundance was calculated using the ΔΔCt method.

### Mitochondrial Membrane Potential (MMP) Measurement

To evaluate mitochondrial viability and function, we monitored changes in mitochondrial membrane potential (MMP) using a 5,5,6,6′-tetrachloro-1,1′,3,3′-tetraethylbenzimi-dazoylcarbocyanine iodide (JC-1) dye (Kulkarni et al., 1998; Sivandzade et al., 2019). Fluorescence intensity was detected using a flow cytometer (FACScan; BD Biosciences, United States) and analyzed using the FACSuite software. The emitted green and red fluorescence was measured using 585-nm (FL2) and 530-nm (FL1) bandpass filters. FL1–FL2 compensation was approximately 4% and FL2–FL1 compensation was 10.6%. Bivariate plots of FL2 vs. FL1 were applied to assess MMP.

### Intracellular ATP Level Measurement

Intracellular ATP level was analyzed using the Bioluminescent Somatic Cell Assay Kit according to the instructions of the manufacturer (Sigma-Aldrich, St. Louis, United States) (Chen et al., 2008). Briefly, viable mitochondria were dissolved to liberate intracellular ATPs, mixed with a substrate and luciferase enzyme, and transferred into a 96-black well plate. Finally, luminescence analysis was conducted using a luminometer.

The article "Resveratrol Improves Mitochondrial Biogenesis Function and Activates PGC-1α Pathway in a Preclinical Model of Early Brain Injury Following Subarachnoid Hemorrhage" was retracted in 2025. Reason: concerns about the images.

### Statistical Analysis

Statistical analysis was conducted using the GraphPad Prism 8.0 software (GraphPad Software Inc., La Jolla, CA, United States). Values were expressed as mean ± SEM. Statistical comparisons between groups were analyzed with one-way ANOVA and Tukey’s test. A *p*-value of <0.05 was considered statistically significant.

## Results

### Resveratrol Restored Neurological Function and Alleviated Cerebral Edema Following SAH

To evaluate the neuroprotective role of RSV on neurological function, neurological scores were recorded 24 and 72 h after SAH as described above. Rats were trained 24 h before SAH. Within 3 days after SAH, there was no statistically significant change between time points in the sham group. No obvious difference was observed between the rats in the SAH group and rats in the SAH + V group at 24 and 72 h (*p* = 0.095, Figure 1C). However, RSV treatment significantly improved motor performance compared with the vehicle-treated rats 24 h after SAH (*p* = 0.0023, Figure 1D). Nevertheless, RSV could not improve motor performance compared to that of the vehicle-treated rats 72 h following SAH. Therefore, 72 h after SAH, the group was not used for the following studies: sacrifice, brain extraction, measurements, and histology. The finding suggested that a 24-h timeframe might be an optimal time point for studying RSV treatment for SAH. Thus, 24 h after SAH the group was used for subsequent studies.

Brain water content was further analyzed to explore the protective role of RSV. As shown in Figure 1B, brain water content was markedly increased in the SAH group when compared with the sham group. No significant difference was observed between the vehicle-treated group and SAH + V group (*p* = 0.1151). Consistent with neurological scores, RSV was successful in ameliorating SAH-induced brain edema than the vehicle-treated group (*p* = 0.021).

### Resveratrol Ameliorated Neuronal Apoptosis Following SAH

To evaluate whether RSV administration could attenuate apoptosis in the inferior temporal cortex 24 h after SAH, TUNEL analysis was performed to assess neuronal apoptosis. As shown in Figure 2, only scattered TUNEL-positive cells were observed in the sham group, whereas the SAH and SAH + V groups displayed numerous apoptotic cells in the temporal cortex up to nearly 36%. However, the apoptosis index in the SAH + RSV group fell to about 22% (Figures 2E,F). We detected the expression of cleaved caspase-3, P53, and Bcl-2 at the protein level. The results indicated that the levels of the antiapoptotic protein Bcl-2 were markedly decreased, and that the levels of the proapoptotic protein P53 and cleaved caspase-3 were notably increased compared with the sham group, whereas these effects were reversed by RSV administration (Figures 2A–D). Collectively, these results demonstrate that RSV treatment possibly abrogated neuronal apoptosis following SAH.

The article "Resveratrol Improves Mitochondrial Biogenesis Function and Activates PGC-1α Pathway in a Preclinical Model of Early Brain Injury Following Subarachnoid Hemorrhage" was retracted in 2025. Reason: concerns about the images.

**FIGURE 2:** Effect of RSV on neuronal apoptosis was evaluated 24 h after SAH. **(A)** Western blot showed pro- and antiapoptotic proteins in the temporal cortex. **(B–D)** Expression of P53, Bcl-2, and cleaved caspase 3 protein levels were standardized to the level of β-actin. **(E)** Representative immunofluorescence images showed that RSV treatment significantly attenuated neuronal apoptosis in the temporal cortex 24 h after SAH. **(F)** The apoptosis index was represented by the percentage of TUNEL-positive cells against neuronal cells. The number of TUNEL-positive neurons was ameliorated by RSV treatment following SAH. Data were presented as mean ± SEM (*n* = 6). Bar = 50 μm. ***p < 0.001 vs. sham group; ^ns^*p* > 0.05 vs. group with SAH; ^##^*p* < 0.01 vs. vehicle-treated group.

### Resveratrol Exerted a Protective Role in Mitochondria

To further elucidate the neuroprotective role of RSV in mitochondria, the expression of mitochondrial apoptosis-related proteins Bax and cytochrome c was examined following SAH. The results showed that the level of mitochondrial Bax protein was increased after SAH, whereas mitochondrial cytochrome c levels were decreased, relative to the sham group (Figures 3C,D,E). However, RSV treatment suppressed mitochondrial translocation of Bax and subsequent cytosolic release of cytochrome c.

**FIGURE 3:** Effect of RSV on mitochondrial function was determined 24 h following SAH. **(A,B)** Representative images of Nissl staining in the temporal cortex showed that RSV could evidently reduce the number of surviving neurons. Arrows point to dead neurons. **(C)** The expression of mitochondrial Bax and cytochrome C in the temporal cortex was detected by Western blot 24 h after SAH. Representative images showed that the relative expression of mitochondrial Bax was decreased, while cytochrome c was restored after RSV administration. Relative protein levels were standardized with respect to COX IV protein **(D,E)**. **(F,G)** The levels of mitochondrial MDA in the temporal cortex were significantly obviously attenuated, and the activities of mitochondrial SOD were significantly increased by RSV treatment. Data were represented as mean ± SEM (*n* = 6). **p < 0.01 vs. sham group; ^ns^*p* > 0.05 vs. group with SAH; ^#^*p* < 0.05 vs. vehicle-treated group.

The article "Resveratrol Improves Mitochondrial Biogenesis Function and Activates PGC-1α Pathway in a Preclinical Model of Early Brain Injury Following Subarachnoid Hemorrhage" was retracted in 2025. Reason: concerns about the images.

To explore the antioxidative effect of RSV after SAH, we determined the production of MDA and SOD in mitochondria. Our results underlined that the activity of SOD was significantly decreased after SAH when compared with the sham group. However, RSV treatment elevated the activity of SOD (*p* = 0.012; Figure 3F). In contrast, SAH insult increased the mitochondrial MDA level, and RSV administration could restore the content of MDA (*p* = 0.016, Figure 3G).

For a better understanding of the comprehensive effects of RSV on EBI following SAH, neuronal survival was further evaluated 24 h post SAH. As shown in Figures 3A,B, RSV significantly increased the proportion of surviving neurons. Taken together, these results suggested that RSV could improve mitochondrial function and promote neuronal survival in the temporal cortex following SAH.

### Resveratrol Administration Ameliorated ROS Induced by SAH

To determine whether the protective role shown by RSV is associated with its antioxidant property, we examined the effect of RSV on ROS production. ROS were detected in the form of superoxide anions following SAH. Intracellular ROS production was detected by DHE fluorescence. As shown in Figure 4, SAH insult significantly (*p* = 0.0061) increased ROS levels showed a significantly higher DHE fluorescence intensity compared with that in the sham group. Interestingly, the total ROS level was significantly reduced by RSV treatment (Figures 4A,B). Then, the mitochondrial ROS content was analyzed by MitoSOX staining. Our results showed that RSV treatment significantly ameliorated the relative level of mitochondrial ROS content (Figure 4C), and this is consistent with the result of DHE fluorescence.

**FIGURE 4:** Effect of RSV on ROS scavenging was evaluated 24 h following SAH. **(A,B)** RSV suppressed the production of intercellular ROS detected by DHE staining. RSV treatment reduced the total ROS content compared with the vehicle group. *n* = 6 per group. **(C)** Mitochondrial ROS was evaluated by MitoSOX staining, and production of mitochondrial ROS was markedly decreased by RSV treatment. *n* = 6 per group. **(D)** Representative images of 8-OHdG by immunofluorescence assay indicated that RSV abrogated the formation of 8-OHdG. *n* = 6 per group. Data were represented as mean ± SEM (*n* = 6). **p < 0.01 vs. sham group; ^ns^*p* > 0.05 vs. group with SAH; ^#^*p* < 0.05 vs. vehicle-treated group.

To further verify the beneficial role of RSV, we determined the expression of 8-hydroxy-2-deoxyguanosine (8-OHdG) by immunofluorescence staining in or around the nucleus following SAH. The observation found that numerous 8-OHdG positive cells with red color were obvious in the SAH and vehicle-treated groups, whereas RSV treatment significantly alleviated the number of 8-OHdG positive cells in the temporal cortex 24 h after SAH (Figure 4D).

The article "Resveratrol Improves Mitochondrial Biogenesis Function and Activates PGC-1α Pathway in a Preclinical Model of Early Brain Injury Following Subarachnoid Hemorrhage" was retracted in 2025. Reason: concerns about the images.

### Resveratrol Promoted PGC-1α Nuclear Translocation

Obtained data demonstrated that RSV markedly increased the activities of antioxidant enzymes induced by SAH. However, the underlying molecular mechanisms remain elusive. PGC-1α plays an essential role in the restoration of mitochondrial function. Accordingly, it is reasonable to hypothesize that RSV might activate PGC-1α, thereby enhancing the restoration of mitochondrial function. We measured the expression level of nuclear PGC-1α and total PGC-1α. Our results suggested that the administration of RSV promoted PGC-1α nuclear translocation compared with the vehicle-treated group (Figure 5A). Additionally, RSV treatment significantly increased the relative protein level of nuclear PGC-1α, while the total PGC-1α level was also upregulated in the SAH + RSV group. This finding suggested that RSV promoted PGC-1α nuclear translocation, thus enhancing its binding activity to promote mitochondrial biogenesis and function.

**FIGURE 5:** Effect of RSV on mitochondrial biogenesis potentially by the PGC-1α pathway was evaluated. **(A,B)** Representative bands of Western blot showed that the level of nuclear PGC-1α and total PGC-1α was elevated by RSV treatment. Relative protein levels of nuclear PGC-1α were standardized to the level of H3. **(C)** Representative immunofluorescence staining of PGC-1α demonstrated that RSV promoted PGC-1α nuclear shuttling. Scale bar = 50 μm; data were represented as mean ± SEM (*n* = 6). **p < 0.01 vs. sham group; ^ns^*p* > 0.05 vs. group with SAH; ^##^*p* < 0.01 vs. vehicle-treated group.

This effect was also confirmed by immunofluorescence staining of PGC-1α. As shown in Figure 5, only a few PGC-1α immunoreactive neurons are seen in the sham group, whereas numerous PGC-1α immunoreactive neurons are seen in the temporal cortex following SAH. These observations demonstrated that SAH promotes PGC-1α nuclear translocation. However, the number of PGC-1α immunoreactive neurons was remarkably increased by RSV treatment compared with the vehicle-treated group. Together, these results suggested that RSV promotes PGC-1α translocation, thereby enhancing the binding ability to downstream proteins.

### Resveratrol Upregulated the Expression of PGC-1α Downstream Factors

Obtained significant evidence indicated that RSV could activate PGC-1α and improve mitochondrial biogenesis and function after SAH. Hence, we speculated that RSV might also regulate downstream factors in the PGC-1α pathway. We measured the expression of NRF1 and TFAM. Our data demonstrated that NRF1 and TFAM were both upregulated following SAH (*p* = 0.0031 and *p* = 0.00056, respectively). However, RSV treatment further promoted the expression of PGC-1α downstream proteins compared with the vehicle-treated group (*p* = 0.0043 and *p* = 0.00025; Figures 6A,B). These results demonstrated that RSV promoted the expression of PGC-1α downstream factors at the protein level by activation of the PGC-1α signaling pathway.

The article "Resveratrol Improves Mitochondrial Biogenesis Function and Activates PGC-1α Pathway in a Preclinical Model of Early Brain Injury Following Subarachnoid Hemorrhage" was retracted in 2025. Reason: concerns about the images.

**FIGURE 6:** Effect of RSV on the expression of PGC-1α downstream proteins was determined after SAH. **(A)** The expression of NRF1 and TFAM was elevated following SAH. Moreover, RSV further upregulated the expression in the temporal cortex after SAH (*n* = 6). **(B)** The ratios of NRF1 and TFAM. Relative protein levels were standardized with respect to β-actin protein. **(C)** MMP. **(D)** Intracellular ATP content. **(E)** mtDNA content. Data were represented as mean ± SEM (*n* = 6). *p < 0.05 and **p < 0.01 vs. sham group; ^ns^*p* > 0.05 vs. group with SAH; ^#^*p* < 0.05 and ^##^*p* < 0.01 vs. vehicle-treated group.

### Mitochondrial Membrane Potential, Intracellular ATP Content, and mtDNA Copy Number

Mitochondrial membrane potential and intracellular ATP content values decreased in the SAH and SAH + vehicle groups, and increased notably after RSV treatment (Figures 6C,D). Furthermore, the mtDNA copy number in the SAH + V group increased compared to the sham group (*p* = 0.035). However, compared to the SAH + V group, the mtDNA copy number was significantly decreased in the SAH + RSV group (Figure 6E). The findings presented above indicated that RSV improved mitochondrial biogenesis in EBI following SAH.

## Discussion

Mitochondria are fundamental in the regulation of the function of neurons. Neurons, which are susceptible to oxidative stress, have fewer endogenous antioxidants than other cells. Extensive evidence demonstrates that mitochondrial dysfunction plays a key role in the development of secondary injury induced by SAH (Shen et al., 2019). SAH increases the ROS levels and impairs the mitochondrial function. Superfluous ROS in mitochondria causes mitochondrial injury, leading to increased ROS synthesis, decreased adenosine triphosphate synthesis, and resulting in the activation of endogenous apoptotic pathway. A recent analysis indicated that mitochondrial dysfunction could be a hallmark for SAH. Consequently, improving mitochondrial biogenesis and function may be a novel beneficial therapeutic target for the treatment of SAH.

In the current study, we investigated the effects of RSV treatment on mitochondrial biogenesis and function *via* activation of the PGC-1α signaling pathway in EBI following SAH. The main findings of this study are as follows: (1) RSV treatment attenuated the mitochondria-dependent apoptosis following SAH; (2) RSV administration reduced redundant ROS production induced by SAH; (3) the PGC-1α signaling pathway was activated by RSV treatment and modulation of PGC-1α nuclear shuttling was promoted following SAH; and (4) SAH-induced oxidative damage, brain edema, and neurological impairment were ameliorated by RSV treatment. These findings indicated for the first time that RSV could promote mitochondrial biogenesis and function against SAH-induced oxidative stress and apoptosis *via* activation of the PGC-1α pathway.

The article "Resveratrol Improves Mitochondrial Biogenesis Function and Activates PGC-1α Pathway in a Preclinical Model of Early Brain Injury Following Subarachnoid Hemorrhage" was retracted in 2025. Reason: concerns about the images.

Resveratrol, a natural phytoalexin product found in grapes and other plants (Dean et al., 2010), is well known for its phytoestrogenic and antioxidant properties (Baur et al., 2006). Recently, studies have demonstrated that RSV could be a promising therapeutic ingredient against various central nervous system diseases (Della-Morte et al., 2009; Zhang et al., 2016a). Previous studies have revealed that RSV has pleiotropic effects, such as antioxidant, anti-apoptotic, and anti-inflammatory, and vasodilatory properties (Della-Morte et al., 2009; Simão et al., 2012; Gatson et al., 2013; Narayanan et al., 2015; Taguchi et al., 2015). RSV treatment can mitigate neuronal apoptosis in numerous types of brain injury, such as cerebral ischemia and SAH, and spinal cord injury (Liu et al., 2011; Zhou X. M. et al., 2014). In this study, we observed that RSV treatment significantly improved the expression of apoptosis-related proteins, such as P53, Bcl2, and cleaved caspase-3, and also promoted neuronal survival in EBI after SAH. RSV treatment alleviated MDA levels and improved the activity of SOD. These results indicated that RSV could attenuate neuronal apoptosis and oxidative damage in EBI following SAH. These findings extend those of previous studies (Zhou X. M. et al., 2014; Zhang et al., 2016b). However, the molecular mechanisms of RSV in EBI have yet to be elucidated.

Neurons appear particularly vulnerable to mitochondrial dysfunction (Chan, 2006). A recent analysis indicated that mitochondrial dysfunction plays an essential role in the pathophysiological process of SAH. Prevention of mitochondrial damage and dysfunction may be a new approach for the treatment of SAH. We speculated that the neuroprotective effects of RSV may be associated with improvement in mitochondrial biogenesis and function, but the exact mechanism remains obscure. The oxidative damage by SAH caused the opening of mitochondrial permeability transition pores (PTPs), leading to increased ROS release to the cytoplasm and resulting in mitochondrial dysfunction. Mitochondrial injury causes overproduction of ROS (Smith et al., 2013), contributing to mitochondrial dysfunction and upsetting the normal balance of endogenous oxidant and antioxidant mechanisms (Smith et al., 2013). Mitochondrial dysfunction leads to oxidative modification of proteins, lipids, and DNA, resulting in excessive ROS release.

The article "Resveratrol Improves Mitochondrial Biogenesis Function and Activates PGC-1α Pathway in a Preclinical Model of Early Brain Injury Following Subarachnoid Hemorrhage" was retracted in 2025. Reason: concerns about the images.

In this study, we assessed the potential effects of RSV on ROS scavenging after SAH. We found that RSV treatment could notably reduce ROS release in the temporal cortex. Therefore, the activity of MDA was decreased and that of SOD is increased by RSV treatment. As a consequence, the mitochondrial proapoptotic protein Bax accumulated in the cytoplasm, while cytochrome c was liberated from the mitochondria, thus triggering the activation of the intrinsic apoptosis pathway (Cahill et al., 2007; Wei et al., 2015), resulting in activation of the mitochondrial-dependent apoptotic pathway, and inducing the sequential activation of the caspase cascades (Park et al., 2004). This series of events causes degradation of DNA and essential proteins and ultimately leads to neuronal apoptosis (Li et al., 1997; Liu et al., 2014). A similar phenomenon was found in this study. Our data showed that RSV significantly ameliorated mitochondrial Bax and restored cytochrome c. These results indicated that the mitochondrial apoptotic pathway was activated following SAH. Moreover, RSV eliminated redundant ROS production generated by mitochondria, erasing free radicals in the mitochondrial root, thus attenuating mitochondrial-dependent apoptosis and improving antioxidative ability. We hypothesize that mitochondrial biogenesis might be accountable for these findings.

Mitochondrial biogenesis is a complicated process that requires coordinated regulation of multiple proteins. Growing data indicate that PGC-1α, NRF-1, and TFAM are responsible for mitochondrial biogenesis (Lagouge et al., 2006). Neuronal mitochondrial biogenesis by itself has been poorly established. PGC-1α, a transcriptional coactivator with pleiotropic functions, plays a pivotal role in mitochondrial biogenesis and function (Wareski et al., 2009). However, the underlying mechanisms by which PGC-1α is activated and mitochondrial biogenesis is upregulated are poorly understood in the rat model of SAH. In this study, we explored the expression of the PGC-1α signaling pathway. We found that the expression of PGC-1α was upregulated by RSV treatment following SAH. RSV treatment also promoted PGC-1α nuclear translocation and PGC-1α downstream genes NRF1 and TFAM were activated. NRF1, bound to the binding sites of the TFAM gene, which regulates the transcription of the mitochondrial genome, together acts on the promoter within the D-loop region of mtDNA, initiating replication and transcription of the mitochondrial genome (Finck and Kelly, 2006; Scarpulla, 2008). The findings indicated that RSV activated PGC-1α and its downstream transcriptional factors (NRF1 and TFAM), which are closely linked to increased mitochondrial biogenesis. Furthermore, increased MMP following RSV treatment suggested the effect on mitochondrial biogenesis post SAH. ATP levels were also analyzed in accordance with alterations of MMP, providing further evidence for the protective effect of RSV on mitochondrial function. Importantly, RSV restored the mtDNA copy number to almost normal levels after SAH. These data suggested that RSV could reverse mitochondrial dysfunction and improve mitochondrial biogenesis following SAH. Increasing evidence suggests that PGC-1α is a powerful regulator of ROS removal because it increases the expression level of numerous ROS-detoxifying enzymes (Valle et al., 2005; St-Pierre et al., 2006). We also found that the activity of the mitochondrial ROS-detoxifying gene SOD was elevated by RSV and that RSV activated PGC-1α. The RSV treatment eliminated the overproduction of ROS originating from mitochondria, improving SAH-mediated mitochondrial impairment and ROS activity. These results showed that the PGC-1α pathway was activated and involved in mitochondrial biogenesis in the early period after SAH. For a better understanding of these neuroprotective effects of RSV following SAH, we further explored SAH-induced brain edema and neurological function 24 h after SAH. Our results indicated that RSV treatment could improve neural survival and neurological impairment.

The article "Resveratrol Improves Mitochondrial Biogenesis Function and Activates PGC-1α Pathway in a Preclinical Model of Early Brain Injury Following Subarachnoid Hemorrhage" was retracted in 2025. Reason: concerns about the images.

There are some limitations to this study. First, an *in vitro* model of SAH should be used to determine whether RSV is involved in neuroprotection against neuronal apoptosis, oxidative stress, and PGC-1α nuclear translocation. Second, a PGC-1α gene knockout mouse model should be used to identify the mitochondria-boosting property of RSV by activation of the PGC-1α pathway. Research in many other associated areas is warranted.

## Conclusion

The findings in this study reveal that RSV treatment could provide neuroprotection in models with SAH by inhibiting mitochondrial-dependent apoptosis, attenuating mitochondria-related ROS release, alleviating mtDNA copy number, and improving antioxidative ability in the temporal cortex. Our data support a previous hypothesis that RSV could improve mitochondrial biogenesis and function after SAH by activating the PGC-1α signaling pathway. The PGC-1α signaling pathway may be a key therapeutic target for future neuroprotective strategies against SAH. A further study should establish the mitochondria-boosting property of RSV in models with neuron SAH *in vitro* and examine underlying mechanisms.

## Data Availability Statement

The original contributions presented in the study are included in the article/supplementary material, further inquiries can be directed to the corresponding author/s.

## Ethics Statement

The animal study was reviewed and approved by the Ethics Committee of The First Affiliated Hospital, Hainan Medical University.

## Author Contributions

JZ conceived the study and drafted the manuscript. ZY, RS, HZ, and WZ performed the experiments. ZC and JZ assisted with data analysis. JZ and JT reviewed and edited the manuscript. All authors read and approved the manuscript.

## Conflict of Interest

The authors declare that the research was conducted in the absence of any commercial or financial relationships that could be construed as a potential conflict of interest.
